The article "Multiple Roles for B-Lymphocytes in Sjogren’s Syndrome" was published in 2016. Journal: J Clin Med.

# Multiple Roles for B-Lymphocytes in Sjogren’s Syndrome

**DOI:** 10.3390/jcm5100087

**Published:** 2016-10-08

**Authors:** Julian Lawrence Ambrus, Lakshmanan Suresh, Ammon Peck

**Affiliations:** 1 Division of Allergy, Immunology and Rheumatology, SUNY at Buffalo School of Medicine, 100 High Street, Buffalo, NY 14203, USA; 2 Immco Diagnostics and the Department of Oral Diagnostic Sciences, SUNY at Buffalo School of Dental Science, Buffalo, NY 14203, USA; lsuresh@immco.com; 3 College of Veterinary Medicine University of Florida, Gainesville, FL 32608, USA; peck@pathology.ufl.edu

**Keywords:** Sjogren’s syndrome, B cells, marginal zone B cells

## Abstract

Sjogren’s syndrome (SS) is a complex heterogeneous autoimmune disease resulting in loss of salivary gland and lacrimal gland function that may include multiple systemic manifestations including lymphoma. Multiple cell types participate in disease pathogenesis. This review discusses evidence for abnormal B cell subpopulations in patients with SS, critical roles of B cells in SS and the status of B cell–directed therapies in the management of patients with SS.

## 1. Introduction

Sjogren’s syndrome (SS) is an autoimmune disease defined by the presence of abnormal salivary and lacrimal gland function commonly characterized by the detection of specific autoantibodies, especially anti-nuclear autoantibodies (ANAs) and Rheumatoid Factor (RF) [1,2,3]. Disease can occur in isolation or as a secondary phenomenon with other autoimmune diseases, such as systemic lupus erythematosus, rheumatoid arthritis, systemic sclerosis, primary biliary cirrhosis and inflammatory bowel disease. In some patients, disease may be restricted to the salivary and lacrimal glands, but in many patients systemic involvement results in pathology of multiple organs and tissues, including the lungs, kidneys and peripheral nervous system [4,5,6], possibly from systemic vasculitis. Of particular interest is the observation that patients with primary SS have a higher incident of associated B cell lymphomas than the general population or patients with other autoimmune diseases [7,8,9]. The presence of autoantibodies, the demonstration of B lymphocytes, and occasional germinal centers in the salivary glands, together with the high incidence of B cell lymphomas, have focused significant attention on the role of B lymphocytes in the pathophysiology of SS.

In support of this overall concept are results arising from studies of mouse models for SS. Perhaps some of the most fascinating and original findings came from the Igμ gene knockout mouse, NOD-IgμNULL [10]. The NOD mouse, a model of secondary Sjögren’s syndrome, exhibits spontaneous and naturally occurring Sjögren’s syndrome in combination with both type 1 diabetes and thyroiditis. In the first study, silencing the Igμ gene in NOD-IgμNULL mice resulted in the complete lack of immunoglobulin production and all clinical manifestations of Sjögren’s syndrome. In the second study, these NOD-IgμNULL mice, when infused with immunoglobulin fractions of sera collected from individual SS patients, resulted in transient stimulation or suppression of salivary flow rates. Taken together, these data strongly point to the importance of mature B cells and their products in the induction and onset of Sjögren’s syndrome in these rodent models, but at the same time reveal the antibodies raised in SS patients have variable activities.

Despite the fundamental knowledge that B lymphocytes play an important role in the development of SS, we are still, decades later, trying to define basic relationships between B lymphocytes and SS disease. In this review we discuss the critical roles for B cells in SS, evidence for abnormal B cell subpopulations in patients with SS, and the status of B cell–directed therapies in the treatment of SS.

## 2. B Cell Subpopulations in Patients with Sjogren’s Syndrome

Studies evaluating the subpopulations of B cells in the peripheral blood of patients with SS have measured decreased numbers of CD27+ memory B cells [11,12,13,14]. Genetic evaluation of these cells has identified increased numbers of mutated Ig transcripts, suggesting a high percentage of the CD27+ cells are IgM memory B cells [12]. These cells demonstrate increased states of activation compared to normal controls that generally would be polyclonal in nature [13]. In contrast, increased numbers of CD27+ memory B cells are noted in the salivary glands of SS patients and these B cells are noted to have undergone antigen-specific selection [15]. The presence of IgM memory B cells has raised the question of T independent B cell selection, an observation that has now led to the identification of increased numbers of marginal zone B (MZB) cells in the peripheral blood and salivary glands of patients with SS [16]. Not surprising then, many of the lymphomas in patients with SS are derived from MZB and these are felt to be indicative of central players in disease pathogenesis per se [17,18,19,20].

Various studies with SS patients have identified increased serum levels and local expression by epithelial cells, B cells and T cells of B cell activating factor (BAFF), a growth and differentiating factor felt to be critical for the activation and survival of B cells [21,22]. Serum BAFF levels correlate with autoantibody production in patients with SS [23]. Furthermore, increased expression of CXCL13 in the salivary glands, a chemokine involved with attracting B cells via binding to the chemokine receptor CXCR5, has been associated with levels of serum autoantibodies and disease activity in SS [24,25,26].

Overall, patients with SS have skewed subpopulations of B cells with both increased antigen-selected memory B cells, IgM memory B cells and CD5 positive B cells [27,28]. The various subpopulations of B cells may have different roles in disease pathogenesis; nevertheless, B cells are clearly involved with autoantibody production, cytokine production, antigen presentation, and possibly various regulatory roles [29,30,31] directing development and onset of SS disease.

## 3. Potential Roles for B Cells in Sjogren’s Syndrome

Studies to evaluate the potential roles for B cells in SS have been performed out of necessity in animal models. Various models have been used, including the MRL/lpr mouse, which carries a mutation in the fas gene and reproduces the human lymphoproliferative syndrome; the NOD mouse, which developed spontaneous diabetes along with SS; the B6.NOD-Aec1Aec2 mouse, which carries genetic regions from the NOD mouse that predisposes C57BL/6J mice to develop SS without diabetes; the BAFF transgenic mouse, which develops proliferative glomerulonephritis along with SS; and the IL-14α transgenic mouse, which develops all the features of SS seen in patients in the same relative time frame, including hypergammaglobulinemia, autoantibodies, salivary and lacrimal gland hypo-function, lymphocytic pneumonitis, renal disease and lymphoma [32,33,34,35,36,37]. Interestingly, increased expression of IL-14α has been noted in patients with SS [36], as well as in MRL/lpr, NOD and B6.NOD-Aec1Aec2 mice (unpublished data).

Several interesting common features have been observed in these animal models. First, increased numbers of MZB and MZB precursors have been noted [38,39,40]. In both BAFF transgenic mice and IL-14α transgenic mice, deletion of MZB results in elimination of all the features of SS [39,41]. Second, salivary gland hypo-function has been noted before lymphocytes are present in the salivary gland, suggesting that the lymphocytes themselves are not directly inducing cellular cytotoxicity [32,36,42]. Third, autoantibodies do not correlate with degree of salivary gland hypo-function [43]. Of additional interest, in the NOD mouse, elimination of IL-4 leads to preservation of salivary gland function despite ongoing lymphocytic infiltration of the salivary glands, again suggesting a dichotomy between lymphocytes in the salivary glands and salivary gland function [44].

In experiments done with NOD mice, salivary gland injury was minimized in NOD mice treated with cobra venom to deactivate complement, suggesting that complement, especially C3, is important in disease pathogenesis [45]. Furthermore, additional studies have indicated that the important pathway is the alternate complement pathway. Complement may be important in SS for many reasons including degradation and presentation of self-antigens, clearance of antigens, and even activations of various cell types, including MZB, which express high levels of CR2 (CD21) [46,47,48]. Additional experiments with this model demonstrated that elimination of both BAFF and CXCL13 resulted in improved salivary gland function, suggesting that B cell migrations and activation/survival of B cells is necessary for salivary gland injury [49].

In the B6.NOD-Aec1Aec2 mouse, elimination of C3 was again shown to dampen the clinical manifestations of SS [40]. Similarly, elimination of the type 1 interferon receptor, or interferon itself, was shown to eliminate multiple features of SS, supporting the notion promoted in human studies on SS that type 1 interferon is a major driver of disease pathogenesis in SS [50,51,52,53].

In the BAFF transgenic mouse, elimination of MZB cells blocks the development of SS, but fails to alter the proliferative glomerulonephritis, suggesting that the nature by which various organs are injured even in the same autoimmune animal are different [41]. Elimination of TNF-α from the BAFF transgenic mice did not influence the development of SS, but did lead to the development of lymphoma, which does not normally occur spontaneously in this model [54]. Various studies have identified increased levels of TNF-α in patients with SS, but it is not known if this cytokine may be playing a protective rather than a destructive role in disease pathogenesis [55]. Unfortunately, a common problem with all clinical studies is the fact that identification of changes in the level of a cytokine does not indicate its role in the disease process, and animal studies are still necessary to rule this out.

In the IL-14α transgenic mouse, several additional observations are of interest. First, eliminating lymphotoxin-alpha (LTα) prevents the development of all the clinical manifestations of SS [43]. MZB spontaneously produces LTα in IL14α transgenic mice, but not in C57BL/6 controls [39]. Eliminating the type 1 interferon receptor has no influence on the early manifestations of SS, submandibular and lacrimal gland injury, but does prevent late manifestations, such as parotid gland and lung injury and lymphoma [37]. This contrasts with the B6.NOD-Aec1Aec2 mouse potentially because there are differences in the cellular abnormalities contributing to the disease pathophysiology between these two models and the effect of type 1 interferon on the immune system is very different depending on the activation state of the cells involved and the chronicity of the antigenic challenge [56,57,58]. Importantly, these variations may be highly indicative of why there are multiple disease phenotypes in the human disease. IL-14α transgenic mice lacking MZB cells fail to produce either LTα or type 1 interferon [39]. Whether MZB cells are the primary source of these cytokines during the evolution of SS is, however, unclear. Interestingly, IL-14α transgenic mice lacking LTα still produce autoantibodies that deposited in the salivary glands, while IL-14α transgenic mice lacking MZB fail to produce the characteristic autoantibodies [39,43]. Clearly, autoantibodies by themselves may not cause salivary and lacrimal gland injury even though a subset of antibodies clearly are important B cell products that may be pathogenic. Furthermore, autoantibodies of different isotypes may have different roles on disease pathogenesis at various stages of disease [59].

Taken together, these studies in mice clearly indicate a central role for MZB cells in SS. They focus on local and systemic features of SS, although limited studies have evaluated dacryoadenitis. However, significant work is needed to understand the various roles that MZB cells play in the disease pathophysiology. Likely cytokine production, in particular LTα and possibly type 1 interferon, is important. MZB cells can be activated via Toll-like receptors as part of the innate immune system to produce various cytokines. In addition, MZB cells have been shown to carry antigens to germinal centers and present antigens to other cell types [48,60]. It is certainly possible that MZB cells are involved with this activity in SS. MZB cells have been shown to react to various self-antigens [61]. They may initiate the response to self-antigen exposure after cellular injury from an environmental toxin/infection. Finally, MZB cells may be directly responsible for autoantibody production or may induce other B cell subpopulations to produce autoantibodies. However, as indicated above, the role of these autoantibodies in the pathogenesis of SS remains unclear.

While autoantibodies are often considered to be the main inducers of local tissue injury, recent studies have raised doubt that this is true. In SS in particular, the functional relevance of autoantibodies to Ro and La, ubiquitous cellular antigens, is unclear. Particular autoantibodies, such as those directed towards muscarinic receptors type 3, have been shown to induce functional changes in vivo and in vitro [62,63], while other autoantibodies, such as anti-salivary gland protein 1, anti-carbonic anhydrase 6 and anti-parotid secretory protein, recognize a variety of salivary gland– and lacrimal gland–specific antigens; however, their full functional activities have not been tested in detail [64,65]. In IL-14α transgenic mice during the early stages of SS, as in patients with early lacrimal gland injury, predominantly IgM antibodies are noted [64], while patients with long-standing SS or secondary SS associated with rheumatoid arthritis, systemic lupus erythematosus (SLE) or systemic sclerosis, have predominantly IgA and to a lesser degree IgG autoantibodies (manuscript in review). This raises the question: are these antibodies merely an epiphenomenon to tissue injury that is occurring, part of a repair process that is attempting to correct the tissue injury, and/or part of a signaling cascade that directs the behavior of multiple cell types? Additional work is necessary to understand this further, as eliminating autoantibodies that are part of a repair process would not be a therapeutic goal. Interestingly, in unpublished data, we have noted that the first lymphocytes that infiltrate the salivary glands in IL-14α transgenic mice produce predominantly IL-10 and TGF-β, suggesting that they may be regulatory cells involved with limiting the extent of the inflammatory process and/or contributing to tissue repair. It should be noted that, in addition to MZB cells, increased numbers of B1 cells are noted in the salivary glands of IL-14α transgenic mice. B1 cells can generate B10 cells that produce IL-10 and these cells are known to inhibit inflammation in autoimmune disease [66,67,68,69].

## 4. B Cell–Targeted Therapies in Sjogren’s Syndrome

The treatment of SS has suffered from many problems: poor understanding of the pathophysiology of the disorder, variability in the disorder itself among different patients, and, most importantly, a delay in the diagnosis of patients with SS. Patients are often diagnosed at a point when there is little healthy glandular tissue remaining in the salivary and lacrimal glands [70,71,72,73,74].

There have been three B cell–targeted therapies evaluated in SS: epratuzumab, an anti-CD22 monoclonal antibody, rituximab, an anti-CD20 monoclonal antibody, and Belimumab, an anti-BAFF monoclonal antibody [75,76,77].

Epratuzumab has been used only in one published, open, labeled study with 16 patients, eight of whom showed some clinical improvement [75]. Whether or not this will be a helpful therapy for SS will require further studies with an expanded patient population.

Similarly, the work with Belimumab is very preliminary. An initial study with 30 patients demonstrated that 60% had improvement in fatigue, but no patient demonstrated improvement in either salivary or lacrimal gland flow. Improvement in certain parameters of B cell activation was achieved in some patients [77,78,79]. Further study is needed to determine whether this will be a beneficial treatment for selected patients with SS.

Rituximab has received the most attention as a therapeutic for SS. It has a much longer history as a therapeutic modality for B cell lymphomas, such as those associated with SS [80,81]. Several trials have been done utilizing rituximab for the treatment of SS [82,83,84,85,86,87], and a recent meta-analysis of these trials concluded that rituximab was weakly effective in improving Schirmer’s tests and salivary gland flow, but had no impact on fatigue or other global measures of well-being [76]. Rituximab was shown to reduce B cell numbers and to normalize the B cell subpopulations seen in the peripheral blood after therapy [88]. Comments made in individual studies identified that treatment early in the course of the disease provided the greatest likelihood of seeing benefit. Furthermore, recent studies have suggested that rituximab may have effects on multiple other cell types besides B cells [89]. A response to rituximab does not necessarily imply that the B cells are critical for disease pathogenesis. At this stage, however, the response to rituximab in the treatment of patients with SS has been marginal, implying the need for further study.

While these B cell–directed therapies show promise, and certainly require further study, there are potential weaknesses that may prevent any of them from becoming the optimal therapy. First of all, rituximab can eliminate all populations of B cells, even though it tends not to impact memory B cells significantly [90]. Beneficial effects would be predicted in eliminating MZB cells, but other B cell populations may have regulatory roles that attempt to limit the severity of SS. In the studies with IL-14α transgenic mice, eliminating MZB cells eliminated the clinical manifestations of SS, but eliminating B1 cells by a Btk knockout resulted in SS disease manifestations occurring earlier and more severely [39]. B1 cells or B1 cell–derived B10 cells are known to play regulatory rolls [91]. Furthermore, as noted above, early production of IgM antibodies may serve to help repair early tissue injury, so eliminating their production may be detrimental. In addition, as noted above, in the IL-14α transgenic mouse, the first lymphocytes infiltrating the salivary glands produce IL-10 and TGF-β. Are these among the cells that should be eliminated? Clearly, more will have to be learned about the roles of different B cell subpopulations in disease pathogenesis at different stages of the disease. More precise tools will be needed to eliminate detrimental B cells and to encourage the proliferation and activity of regulatory B cells.

## 5. Conclusions

Studies evaluating patients with SS, as well as various animal models for SS, demonstrate abnormal B cell subpopulations, activities and products as central to the pathophysiology of SS as it progresses from a localized disease of the salivary and lacrimal glands initiated by an innate immune response to a systemic disease involving both the innate and adaptive immune system that can undergo lymphomagenesis. MZB cells appear to be key players in this disease, while other B cell subpopulations may play a variety of other roles. Further research is necessary to understand the roles of these critical cells so that more specific and efficacious therapies can be developed.
